The article "Design of a Regional Economic Forecasting Model Using Optimal Nonlinear Support Vector Machines" was retracted in 2023. Reasons: unreliable results or conclusions; concerns about the data; concerns about the results or conclusions; concerns about the peer review.

# Design of a Regional Economic Forecasting Model Using Optimal Nonlinear Support Vector Machines

**DOI:** 10.1155/2022/2900434

**Published:** 2022-01-30

**Authors:** Tong Zhang

**Affiliations:** Department of Artificial Intelligence, Chongqing College of Finance and Economics, Yongchuan 402160, Chongqing, China

## Abstract

Forecasting regional economic activity is a progressively significant element of regional economic research. Regional economic prediction can directly assist local, national, and subnational policymakers. Regional economic activity forecast can be employed for defining macroeconomic forces, such as prediction of stock market and cyclicality of national labor market movement. The recent advances of machine learning (ML) models can be employed to solve the time series prediction problem. Since the parameters involved in the ML model considerably influence the performance, the parameter tuning process also becomes essential. With this motivation, this study develops a quasioppositional cuckoo search algorithm (QOCSA) with a nonlinear support vector machine (SVM)-based prediction model, called QOCSO-NLSVM for regional economic prediction. The goal of the QOCSO-NLSVM technique is to identify the present regional economic status. The QOCSO-NLSVM technique has different stages such as clustering, preprocessing, prediction, and optimization. Besides, the QOCSO-NLSVM technique employs the density-based clustering algorithm (DBSCAN) to determine identical states depending upon the per capita NSDP growth trends and socio-economic-demographic features in a state. Moreover, the NLSVM model is employed for the time series prediction process and the parameters involved in it are optimally tuned by the use of the QOCSO algorithm. To showcase the effective performance of the QOCSO-NLSVM technique, a wide range of simulations take place using regional economic data. To determine the current economic situation in a region, the QOCSO-NLSVM technique is used. The simulation results reported the better performance of the QOCSO-NLSVM technique over recent approaches. The QOCSO-NLSVM technique generated effective results with a minimal mean square error of 70.548 or greater. Astonishingly good results were obtained using the QOCSO-NLSVM approach, which had the lowest root mean square error (RMSE) of 8.399.

## 1. Introduction

The forecasting method predicts future value based on a provided time series data set by making assumptions on future trends and estimating historical data. This is employed for several regions of the decision-making process, like industrial process control, risk management, operations management, demography, and economics [1]. Forecasting is an important problem spanning several domains, involving finance, social science, government, economics, environmental science, politics, medicine, business, and industry. The forecasting problem is categorized as long-term, short-term, and medium-term [2, 3].

The article "Design of a Regional Economic Forecasting Model Using Optimal Nonlinear Support Vector Machines" was retracted in 2023. Reasons: unreliable results or conclusions; concerns about the data; concerns about the results or conclusions; concerns about the peer review.

Forecasting regional economic activity is an essential component of regional economic study. The regional economic prediction could directly assist business executives, local, subnational, and national policymakers. These two business executives and policymakers require precise prediction of key economic aggregates, namely, employment, output, and income for medium-long term planning purposes [4]. Regional economic activity forecasts have been employed for explaining macroeconomic forces, involving the cyclicality of national labour market movements and predicting the stock market. Further, multinational agencies and international investors engaged in megaprojects at a regional level also require precise predictions for investment planning reasons [5]. When there is no paucity of research on predicting national economic indicators, the research on regional economic prediction is limited for innovative economies, and in the case of developing nations, zilch [6]. Problems with short-term forecasting are those that deal with predicting events in a shorter period of time (months, days, and weeks). Forecasting concerns could go much beyond 1-2 years into the future, with medium-term forecasts extending into the future as well.

The forecasting method connected to economic problems is utilized for predicting economic variables in several countries. The industry volatility prediction, critical to several important problems in business [7], and the prediction of the unemployment rates that define the country's economic and social development [8, 9]. Radial basis function networks (RBF) and backpropagation are the ANN architectures that are used in economic fields. The artificial neural networks (ANN) technique was broadly examined in economic analysis. The ANN is a computation system that is performed in hardware or software under the effect of biological studies about the human brain. Several authors admit that the ANN method is the better performing nonlinear analysis technique as well as one of the best predictors [10]. The ANN architecture employed in economic fields is radial basis function networks (RBF) and backpropagation.

This study designs a quasioppositional cuckoo search algorithm (QOCSA) with a nonlinear support vector machine (SVM)-based prediction model, called QOCSO-NLSVM for regional economic prediction. The QOCSO-NLSVM technique involves the design of the density-based clustering algorithm (DBSCAN) to determine the identical states depending upon the per capita NSDP growth trends and socioeconomic-demographic features in a state. Besides, the NLSVM model is elected for the time series prediction process and the parameters involved in it are optimally tuned by the use of the QOCSO algorithm. The experimental validation of the QOCSO-NLSVM technique and the results are examined in various aspects.

The article "Design of a Regional Economic Forecasting Model Using Optimal Nonlinear Support Vector Machines" was retracted in 2023. Reasons: unreliable results or conclusions; concerns about the data; concerns about the results or conclusions; concerns about the peer review.

The rest of the research work is organized as follows.  Section 2 provides the recently developed techniques, Section 3 elaborates the QOCSO-NLSVM technique. Then, Section 4 provides the performance validation, and Section 5 concludes the outcomes of the research.

## 2. Literature Review

Mishra and Ayyub [11] introduced a DL architecture in which the hierarchical clustering analysis (HCA) is utilized for predicting growth. The presented method comprises HCA and DTW techniques that are initially applied for identifying similar socio-economic-demographic features within a provided state and similar states according to per capita NSDP growth trends, to create a fine-tuned training dataset for predicting all the states' NSDP per capita growth. Lv et al. [12] developed a LightGBM-enhanced LSTM for realizing stock price prediction, and LSTM is utilized for predicting the Shenzhen and Shanghai 300 indexes, respectively. The simulation result shows that the LightGBM-LSTM has a better capacity for tracking stock index price trends and the maximum prediction performance, and its effects are superior to the RNN and GRU methods. LightGBM-optimized LSTM for short-term stock price forecasting. To compare its performance with other deep network models such as RNN (recurrent neural network) and GRU (gated recurrent unit), the LightGBM-LSTM, RNN, and GRU are used to predict the Shanghai and Shenzhen 300 indexes, respectively. Experiment results demonstrate that the LightGBM-LSTM has the highest prediction accuracy and the best ability to track stock index price trends.

Zhu et al. [13] designed an experiment whose samples originated from information on 7 quoted core enterprises (CEs) and 46 quoted SMEs in the Chinese security markets. Matta et al. [14] introduced a relative assessment of various prediction techniques using the Gaussian process regression and ANN methods (MLP and RBFNN). Two real-time datasets were utilized for evaluating the prediction method presented in the study. These datasets were normalized to values amongst one and zero. Next, the data training was implemented and, when it was constructed, a system was utilized for generating the predictions. Therefore, observations were made to validate how precisely the fitted method predicts the values.

The article "Design of a Regional Economic Forecasting Model Using Optimal Nonlinear Support Vector Machines" was retracted in 2023. Reasons: unreliable results or conclusions; concerns about the data; concerns about the results or conclusions; concerns about the peer review.

Chatzis et al. [15] integrated distinct ML methods that were proposed with daily currency, stock, and bond data from thirty-nine countries that cover a larger spectrum of economies. It especially leverages the advantages of a sequence of techniques that includes Classifier Trees, SVM, NN, RF, XGBoost, and DNN. Sun et al. [16] verified the cointegration relationships and Granger causality between tourist arrivals in Beijing and the internet search index. This experiment result suggests that compared to standard methods, the presented KELM model that incorporates tourist volume series with Google and Baidu Index could significantly enhance the prediction performances in terms of robustness analysis and forecasting accuracy.

## 3. The Proposed Model

In this study, an effective QOCSO-NLSVM technique has been developed for regional economic prediction. The QOCSO-NLSVM technique encompasses several subprocesses, namely, DTW-based preprocessing, DBSCAN-based clustering, NLSVM-based prediction, and QOCSO-based parameter optimization.  Figure 1 illustrates the overall working process of the QOCSO-NLSVM technique.

### 3.1. Data Preprocessing

One of the primary methods used to capture similarities among two regions, or among pairs of factors within a provided region according to time-series data is named dynamic time warping (DTW). DTW is an effective method utilized for learning similarity based on distance between two sequences that might differ in speed and quantifying time-based similarities among any two pairs. Generally, DTW is an ML method which estimates an optimum match between two provided sequences with some restrictions. The sequence is “warped” nonlinearly in the time dimension to define measures of their similarity, independent of nonlinear variation in the time dimension. The Euclidean distance uses the distance among every pair of the time series and compares it with the Euclidean distance. Simultaneously, the DTW searches for optimal alignments among the two-time series. Furthermore, all the points are utilized for comparing the points to make the best possible alignments among the two-time series according to their distance matrix.

### 3.2. Process Involved in the DBSCAN Technique

DBSCAN might find distinct clusters based on the assessed density distribution. It could recognise structured groupings without knowing their numbers. The following illustrates DBSCAN's basic premise: DBSCAN finds each point in the neighbourhood of a random unvisited point *p*, where it denotes the neighbourhood's maximum radius from *p*. To construct a dense zone, MinPts is the minimum number of points required. When MinPts is in the distance, *p* denotes a core point. When *p* is a core point, all points in its vicinity are grouped together. DBSCAN detects each density-reachable point in the cluster and adds it to a comparable cluster. When a point *q* is densely approachable from other core points but its neighbourhood is less than MinPts, it is a border point. An outlier or noisy point is one that is not accessible from other locations. DBSCAN achieves clustering by extracting clusters consecutively. Rep until no more density-reachable points are identified, and the final cluster is reached. DBSCAN divides a set of points into low-noise border points and high-density. The purpose of DBSCAN is to identify identical states based on a state's per capita NSDP growth trends and socioeconomic-demographic characteristics. DBSCAN was capable of detecting a variety of clusters based on the density distribution that was assessed. The DBSCAN methodology permits the calculation of identical states based on per capita income.

The article "Design of a Regional Economic Forecasting Model Using Optimal Nonlinear Support Vector Machines" was retracted in 2023. Reasons: unreliable results or conclusions; concerns about the data; concerns about the results or conclusions; concerns about the peer review.

Assume two points *x* and *y*, *d*(*x*,  *y*) represent the similarities among them, Γ*ε* (*x*) denotes the *ε*-neighbourhood of *x*, in which Γ*ε* (*x*) = {*y*  ∈  *V|d*(*x*,  *y*)  ≤  *ε*} · *ρ*(*x*) = |Γ*ε*(*x*)|  indicates the density value of *x*:

(1) $$\begin{array}{c} S\left(x\right)=\left\{\begin{array}{cc} 1, & \text{core point with }\rho \left(x\right)\geq \text{MinPts},\\ 0, & \text{border point with }1<\rho \left(x\right)<\text{MinPts},\\ -1, & \text{noise with }\rho \left(x\right)=1. \end{array}\right. \end{array}$$

### 3.3. Structure of the NLSVM Model

During the prediction process, the NLSVM model receives the clustered data as input to predict the output. Assume a trained set {*x*_*k*_, *y*_*k*_}_*k*=1_^*N*^ with input data *x*_*k*_ ∈ *ℝ*^*n*^ and respective binary class label *y*_*k*_ ∈ {−1,  +1}, the SVM classification initiates from the subsequent assumption:

(2) $$\begin{array}{c} \left\{\begin{array}{cc} w^{T}\varphi \left(x_{k}\right)+b\geq +1, & \;i\text{f }y_{k}=+1,\\ w^{T}\varphi \left(x_{k}\right)+b\leq -1, & \;i\text{f }y_{k}=-1. \end{array}\right. \end{array}$$

That is equal to

(3) $$\begin{array}{c} y_{k}\left[w^{T}\varphi \left(x_{k}\right)+b\right]\geq 1,\;k=1,\ldots ,\;N. \end{array}$$

Now, the nonlinear function *φ*(*·*) : *ℝ*^*n*^⟶*ℝ*^*n*_*h*_^ maps the input space to a high-dimensional feature space. It is noteworthy that the *n*_*h*_ dimension of this space is determined in an implicit manner (it is an infinite dimension). The *b* represent a bias as follows:

(4) $$\begin{array}{c} y\left(x\right)=\text{sign}\left[w^{T}\varphi \left(x\right)+b\right]. \end{array}$$

But, at the same time, it is never evaluated in this form. One determines the optimization issue:

(5) $$\begin{array}{c} \;\min\;J\left(w,\;\xi \right)=\frac{1}{2}w^{T}w+c\overset{N}{\underset{k=1}{\sum }}\xi_{k}, \end{array}$$

subjected to

(6) $$\begin{array}{c} \left\{\begin{array}{c} y_{k}\left[w^{T}\varphi \left(x_{k}\right)+b\right]\geq 1-\xi_{k},\;\;k=1,\;\ldots ,N,\\ \xi_{k}\geq 0,\;\;k=1,\;\ldots ,N. \end{array}\right. \end{array}$$

To permit misclassification in the subset of inequalities (because of overlapping distribution), the minimalization of ‖*w*‖_2_ corresponds to a maximalization of the margin among the two classes. *c* indicates a positive real constant and must be taken into account as a tuning parameter. The Lagrangian can be expressed as follows [17]:

(7) $$\begin{array}{c} L\left(w,\;b,\xi ;\alpha ,\;\nu \right)=J\left(w,\xi \right)-\overset{N}{\underset{k=1}{\sum }}\alpha_{k}\left\{y_{k}\left[w^{T}\varphi \left(x_{k}\right)+b\right]-1+\xi_{k}\right\}-\overset{N}{\underset{k=1}{\sum }}\nu_{k}\xi_{k}. \end{array}$$

The Lagrange multiplier is *α*_*k*_ ≥ 0, *ν*_*k*_ ≥ 0,  (*k*=1,  *N*).  Figure 2 depicts the SVM hyperplane. It is familiar from the optimization concept that the solutions are considered by the saddle points of the Lagrangian:

(8) $$\begin{array}{c} \underset{\alpha ,\;v}{\max}\underset{w,\;b,\;\xi \;}{\min}ℒ\left(w,\;b,\;\xi ;\alpha ,\;\nu \right). \end{array}$$

One attains

(9) $$\begin{array}{c} \left\{\begin{array}{c} \frac{\partial L}{\partial w}=0\;⟶\;w=\overset{N}{\underset{k=1}{\sum }}\alpha_{k}y_{k}\varphi \left(x_{k}\right),\\ \frac{\partial L}{\partial b}=0\;⟶\;\overset{N}{\underset{k=1}{\sum }}\alpha_{k}y_{k}=0,\\ \frac{\partial L}{\partial \xi_{k}}=0\;⟶\;0\leq \alpha_{k}\leq c,\;\;k=1,\;\ldots ,N. \end{array}\right. \end{array}$$

By substituting *w* in the Lagrangian, one attains the subsequent binary problems (in the Lagrange multiplier *α*), i.e., the quadratic programming problems:

(10) $$\begin{array}{c} \underset{\alpha }{\max}Q\left(\alpha \right)=-\frac{1}{2}\overset{N}{\underset{k,l=1}{\sum }}y_{k}y_{l}K\left(x_{k},\;x_{l}\right)\alpha_{k}\alpha_{l}+\overset{N}{\underset{k=1}{\sum }}\alpha_{k}. \end{array}$$

Thus,

(11) $$\begin{array}{c} \left\{\begin{array}{c} \overset{N}{\underset{k=1}{\sum }}\alpha_{k}y_{k}=0,\\ 0\leq \alpha_{k}\leq c,\;\;k=1,\;\ldots ,N. \end{array}\right. \end{array}$$

Now *w* and *φ*(*x*_*k*_) are not estimated. According to the Mercer condition, one takes a kernel as

(12) $$\begin{array}{c} K\left(x_{k},\;x_{l}\right)=\varphi {\left(x_{k}\right)}^{T}\varphi \left(x_{l}\right). \end{array}$$

Lastly, in binary space, the nonlinear SVM classifiers become

(13) $$\begin{array}{c} y\left(x\right)=\text{sign}\left[\overset{N}{\underset{k=1}{\sum }}\alpha_{k}y_{k}K\left(x,\;x_{k}\right)+b\right]. \end{array}$$

*α*_*k*_ is a positive real constant, and *b* is a real constant. The nonzero Lagrange multiplier *α*_*k*_ is known as support value. The respective data point is known as a support vector and is placed near the decision boundary. This is the data point that contributes to the classification method. The bias *b* follows from the KKT condition that isn't considered further.

The article "Design of a Regional Economic Forecasting Model Using Optimal Nonlinear Support Vector Machines" was retracted in 2023. Reasons: unreliable results or conclusions; concerns about the data; concerns about the results or conclusions; concerns about the peer review.

Various selections for the kernel *K*(*·*, *·*) are feasible.

- *K*(*x*, *x*_*k*_)=*x*_*k*_^*T*^*x* (linear SVM)
- *K*(*x*, *x*_*k*_)=(*x*_*k*_^*T*^*x*+1)^*d*^ (polynomial SVM of degree *d*)
- *K*(*x*, *x*_*k*_)=  exp   {−‖*x* − *x*_*k*_‖_2_^2^/*σ*^2^} (RBF kemel)
- *K*(*x*, *x*_*k*_)=tanh(*κx*_*k*_^*T*^*x*+*θ*) (MLP SVM)

The Mercer conditions hold for each *σ* value in the RBF case, but not for each feasible selection of *κ*, *θ* in the MLP case. In the case of an MLP or RBF kernel, the amount of hidden units corresponds to the number of support vectors.

### 3.4. Design of the QOCSO Algorithm for Parameter Tuning

For optimally tuning the weight values of the NLSVM model, the QOCSO algorithm is utilized. The CSO algorithm is assumed as a metaheuristic technique that was primarily established by Yang and Deb [18]. Actually, this CSO method simulates the breeding performance of cuckoo birds that are supposed to be a type of parasitism. The cuckoo birds place their eggs from other nests and play to host the egg. The cuckoo birds attempt for raising the hatch possibility of their individual eggs by generating them the same as the host egg with respect to size, shape, and colour, or by throwing other native eggs (Algorithm 1).

In the CSO technique, cuckoo eggs from distinct nests signify the generation of candidate solutions to optimize problems. Actually, the search starts with particular nests with a solution per nest. This solution was progressed dependent upon the model of cuckoo's recognition (*p*) which was inspired by eliminating the solution of exchanging novel ones.

In the CSO method, a random walk was utilized dependent upon the Lévy flight distribution for producing novel candidate solutions (cuckoos) in the present one as follows:

(14) $$\begin{array}{c} {\text{cuckoo}}_{i}^{\left(t+1\right)}={\text{cuckoo}}_{i}^{\left(t\right)}+a⊕\text{Levy}\left(\lambda \right), \end{array}$$

where cuckoo_*i*_^(*t*+1)^ refers the *i*^th^ cuckoo value *t*. An *a* and *λ* stand for step sizes (generally fixed to one) and coefficients (1 < *λ* < 3) correspondingly. A number of novel solutions were created in the optimum present ones by Lévy walks for performing a local search with self‐improvement [19]. Besides, a few novel solutions were created away from the optimum present ones. This reduces the chance of getting stuck from the local minimal and ensures the searching ability. The CS execution also makes sure elitism as the optimal nest is retained under the iteration.

The article "Design of a Regional Economic Forecasting Model Using Optimal Nonlinear Support Vector Machines" was retracted in 2023. Reasons: unreliable results or conclusions; concerns about the data; concerns about the results or conclusions; concerns about the peer review.

The OBL method was proposed with the aim of decreasing the computation time and improving the ability of various EAs [20]. Therefore, the comparisons among an arbitrary CSO algorithm and its opposite might result in the global optimal with fast convergence rates. Further, the quasiopposite number and showed that it is nearer to the optimum solution when compared to the opposite number. Therefore, the population initialization of this method is created according to the QOBL concept. For arbitrary number *χ* ∈ [*a*, *b*] , its opposite number *χ*_0_ is represented as follows:

(15) $$\begin{array}{c} x_{0}=a+b-x. \end{array}$$

However, the opposite point for multidimensional searching space (dimension) is determined by the following equation:

(16) $$\begin{array}{c} x_{0}^{i}=a^{j}+b^{i}-x^{i},\;\;i=1,2,\;\ldots ,d. \end{array}$$

The quasiopposite no. *x*_*qo*_ of arbitrary no. *χ* ∈ [*a*, *b*] is represented as follows [21]:

(17) $$\begin{array}{c} x_{qo}=\text{rand}\left(\frac{a+b}{2},x_{0}\right). \end{array}$$

Likewise, the quasiopposite point for multidimensional searching space (*d* dimension) is determined by the following equation:

(18) $$\begin{array}{c} x_{qo}^{i}=\text{rand}\left(\frac{a^{i}+b^{i}}{2},x_{0}^{i}\right). \end{array}$$

For obtaining an objective function that could generalize the SVM outcome with no utilization of testing data, the cross validation approach is utilized. The cross validation process partitions the training dataset *D* randomly into *S*  different parts {*G*_*s*_,   *s* = 1,   …,  *S*}, and utilizes (*S* − 1) parts to train the model and to test the model. This process gets iterated for *S* times by varying the lasting parts, and the generalization efficiency can be determined by the use of MSE (mean squared error) over every test result.

(19) $$\begin{array}{c} MSE_{CV}=\frac{1}{N}\overset{S}{\underset{s=1}{\sum }}\underset{i\in G_{s}}{\sum }{\left(y_{i}-f\left(x_{i}|\theta_{s}\right)\right)}^{2}, \end{array}$$

where *G*_*s*_ indicates the *s*-th part for the testing process and  *θ*_*s*_ signifies the solution vector attained at the time of training process.

## 4. Performance Evaluation and Discussion

The performance validation of the QOCSO-NLSVM technique using the economic data from the Niti Aayog website and the Reserve Bank of India were inspected. The data includes several features such as fiscal deficits, revenue deficits, interest payments, capital expenditure, nominal NSDP series, social sector expenditure, electricity generation, infrastructure projects, per capita NSDP at factor cost (at constant prices), per capita NSDP, number of factories, state-wise fixed capital, sectoral growth rate, and pattern of land use.  Table 1 and Figure 3 investigate the actual and predicted result analysis of the QOCSO-NLSVM technique over distinct years. The results portrayed that the QOCSO-NLSVM technique predicted the economic status much closer to the actual value under all runs.

The article "Design of a Regional Economic Forecasting Model Using Optimal Nonlinear Support Vector Machines" was retracted in 2023. Reasons: unreliable results or conclusions; concerns about the data; concerns about the results or conclusions; concerns about the peer review.

For instance, with an actual value of 16855.712, the QOCSO-NLSVM technique has attained predicted values of 16854.72, 16784.71, 16716.72, 16799.72, and 16851.73 under runs 1–5, respectively. At the same time, with the actual values of 18176.991, the QOCSO-NLSVM system has accomplished forecasted values of 18110.02, 18125.98, 18285.98, 18211.01, and 18294.03 under runs 1–5 correspondingly. Furthermore, with the actual values of 21138.478, the QOCSO-NLSVM method has achieved forecasted values of 21028.50, 21282.49, 21097.47, 21184.48, and 21098.48 under runs 1–5 correspondingly. Moreover, with the actual values of 22231.951, the QOCSO-NLSVM algorithm has reached predicted values of 22310.96, 22177.95, 22379.96, 22330.96, and 22374.97 under runs 1–5 correspondingly.

A brief MSE analysis of the QOCSO-NLSVM technique under various runs and years is provided in Figure 4 and Table 2. The experimental values are denoted by the QOCSO-NLSVM technique, which has resulted in an effective outcome with minimal MSE values. For instance, in the year 2012, the QOCSO-NLSVM technique resulted in at least MSE of 70.997, 138.996, 55.994, 3.979, and 0.995, respectively. Simultaneously, in the year 2015, the QOCSO-NLSVM system has resulted in a minimum MSE of 51.009, 108.987, 34.014, 117.037, and 66.972 correspondingly. Simultaneously, in the year 2018, the QOCSO-NLSVM model has resulted in a minimum MSE of 144.010, 41.006, 46.005, 39.996, and 109.978 correspondingly. Likewise, in the year 2020, the QOCSO-NLSVM method has resulted in a minimum MSE of 54.003, 148.011, 99.014, 143.021, and 79.009 correspondingly.

A brief RMSE analysis of the QOCSO-NLSVM method over many years and runs has been demonstrated in Table 3 and Figure 5. The experiment values showed that the QOCSO-NLSVM method has resulted in outstanding results with the smallest RMSE value. For example, in the year 2012, the QOCSO-NLSVM system resulted in a minimal RMSE of 8.426, 22.790, 7.483, 1.995, and 0.997 correspondingly. Concurrently, in the year 2015, the QOCSO-NLSVM approach resulted in a minimum RMSE of 7.142, 10.440, 5.832, 10.818, and 8.184 correspondingly. Simultaneously, in the year 2018, the QOCSO-NLSVM process has resulted in the smallest RMSE of 12.000, 6.404, 6.783, 6.324, and 10.487 correspondingly. Likewise, in the year 2020, the QOCSO-NLSVM method has resulted in a minimal RMSE of 7.349, 12.166, 9.951, 11.959, and 8.889 correspondingly.

The article "Design of a Regional Economic Forecasting Model Using Optimal Nonlinear Support Vector Machines" was retracted in 2023. Reasons: unreliable results or conclusions; concerns about the data; concerns about the results or conclusions; concerns about the peer review.

Table 4 presents a full comparison study of the QOCSO-NLSVM approach.

Figure 6 offers the MSE analysis of the QOCSO-NLSVM technique with recent methods. The figure shows that the LSTM and ARIMA models have obtained poor performance with a higher MSE of 149.997 and 142.235, respectively. Similarly, the GRU and multivariate LSTM models reached a moderate MSE of 128.357 and 95.184, respectively. However, the QOCSO-NLSVM technique has accomplished effective outcomes with a minimal MSE of 70.548.

Figure 7 provides the RMSE of the QOCSO-NLSVM model with current methodologies. The abovementioned figure exhibits that the ARIMA and LSTM systems have gained poor performance with a high RMSE of 11.926 and 12.247 correspondingly. Simultaneously, the multivariate LSTM and GRU methods have attained reasonable RMSE of 9.756 and 11.329, respectively. But, the QOCSO-NLSVM process has gained remarkable results with the smallest RMSE of 8.399.

From the abovementioned figures, it is ensured that the QOCSO-NLSVM model is an effective regional economic prediction method over the other existing techniques.

## 5. Conclusion

In this research, a proposed QOCSO-NLSVM technique has been developed for regional economic prediction. The QOCSO-NLSVM technique encompasses several subprocesses, namely, DTW based preprocessing, DBSCAN-based clustering, NLSVM-based prediction, and QOCSO-based parameter optimization. The use of the DBSCAN model enables the computation of identical states depending upon the per capita NSDP growth trends and socioeconomic-demographic features in a state. In addition, the application of the QOCSO algorithm helps to properly select the parameter values and thereby reaches the maximum predictive outcomes. The QOCSO-NLSVM technique is used to discover identical states based on per capita NSDP growth trends and socioeconomic-demographic characteristics in a state. QOCSO-NLSVM is used to run a variety of simulations on regional economic data and is also used to assess a region's present economic position. The experimental validation of the QOCSO-NLSVM technique and the results are examined in various aspects. The comparative analysis revealed the enhanced outcomes of the QOCSO-NLSVM technique over the recent approaches. With a minimum MSE of 70.548, the QOCSO-NLSVM approach produced effective results. The QOCSO-NLSVM technique had remarkable results, achieving the lowest root mean square error (RMSE) of 8.399. In the future, advanced DL models can be used to improve the overall prediction outcomes.

The article "Design of a Regional Economic Forecasting Model Using Optimal Nonlinear Support Vector Machines" was retracted in 2023. Reasons: unreliable results or conclusions; concerns about the data; concerns about the results or conclusions; concerns about the peer review.

## Figures and Tables

**Figure 1:** System architecture of the QOCSO-NLSVM method.

**Figure 2:** SVM hyperplane.

**Figure 3:** Actual and prediction analysis of the QOCSO-NLSVM technique.

**Figure 4:** MSE analysis of the QOCSO-NLSVM technique with distinct runs.

**Figure 5:** RMSE analysis of the QOCSO-NLSVM technique with distinct runs.

**Figure 6:** MSE analysis of the QOCSO-NLSVM technique with existing approaches.

**Figure 7:** RMSE analysis of the QOCSO-NLSVM technique with existing approaches.

**Algorithm 1:** Pseudocode of the CSO algorithm.

**Table 1:** Actual and predicted analysis of the QOCSO-NLSVM technique with varying years.

Years	Actuals	Run: 1	Run: 2	Run: 3	Run: 4	Run: 5
2012	16855.712	16854.72	16784.71	16716.72	16799.72	16851.73
2013	17037.957	17134.99	17056.94	17098.97	17102.96	17028.95
2014	17675.816	17767.80	17563.80	17820.81	17781.81	17734.82
2015	18176.991	18110.02	18125.98	18285.98	18211.01	18294.03
2016	18860.411	18924.41	18782.41	18806.42	18750.44	18970.43
2017	19999.445	19966.48	20106.45	19960.45	19859.44	19874.43
2018	21138.478	21028.50	21282.49	21097.47	21184.48	21098.48
2019	21730.776	21822.77	21680.80	21651.76	21680.76	21627.80
2020	22231.951	22310.96	22177.95	22379.96	22330.96	22374.97

**Table 2:** MSE analysis of the QOCSO-NLSVM technique with distinct runs.

Years	Run: 1	Run: 2	Run: 3	Run: 4	Run: 5
2012	70.997	138.996	55.994	3.979	0.995
2013	18.987	61.017	65.000	9.006	97.028
2014	112.011	144.993	105.997	59.004	91.982
2015	51.009	108.987	34.014	117.037	66.972
2016	77.999	53.994	109.975	110.019	64.000
2017	107.001	38.997	140.001	125.018	32.967
2018	144.010	41.006	46.005	39.996	109.978
2019	49.977	79.014	50.013	102.978	91.997
2020	54.003	148.011	99.014	143.021	79.009
Average	76.222	90.557	78.446	78.895	70.548

**Table 3:** RMSE analysis of the QOCSO-NLSVM technique with distinct runs.

Years	Run: 1	Run: 2	Run: 3	Run: 4	Run: 5
2012	8.426	11.790	7.483	1.995	0.997
2013	4.357	7.811	8.062	3.001	9.850
2014	10.584	12.041	10.296	7.681	9.591
2015	7.142	10.440	5.832	10.818	8.184
2016	8.832	7.348	10.487	10.489	8.000
2017	10.344	6.245	11.832	11.181	5.742
2018	12.000	6.404	6.783	6.324	10.487
2019	7.069	8.889	7.072	10.148	9.592
2020	7.349	12.166	9.951	11.959	8.889
Average	8.456	9.237	8.644	8.177	7.926

**Table 4:** Comparative analysis of the QOCSO-NLSVM technique with existing approaches.

	MSE	RMSE
LSTM	149.997	12.247
ARIMA	142.235	11.926
GRU	128.357	11.329
Multivariate LSTM	095.184	09.756
QOCSO-NLSVM	070.548	08.399

## Data Availability

No data were used to support this study.
